This article has been retracted.

# Tetramethylpyrazine Inhibits the Proliferation and Invasion of Glioma Cells by Regulating the UBL7-AS1/miR-144-3p Pathway

**DOI:** 10.1155/2022/5261285

**Published:** 2022-08-22

**Authors:** Rui Liang, Guofeng Zhang, Wenhua Xu, Weibing Liu, Youjia Tang

**Affiliations:** Department of Neurosurgery, The First Hospital of Jiujiang City, Jiujiang, Jiangxi 332000, China

## Abstract

This work aims to investigate the effects of tetramethylpyrazine (TMP) on the proliferation, migration, and invasion of glioma cells and to analyze the regulation mechanism of TMP on the long noncoding RNA UBL7-AS1/miR-144-3p pathway. Glioma cell line and normal astrocytes were collected. The expression of UBL7-AS1 was detected by real-time PCR. The glioma cells were overexpressed with UBL7-AS1. CCK-8 and Transwell assays were used to detect cell proliferation and cell invasion ability, respectively. Bioinformatics was adopted to predict the possible regulatory mechanisms of UBL7-AS1. The dual luciferase reporter gene was applied to verify the regulatory effect of RNA UBL7-AS1 with miR-144-3p. TMP inhibited the proliferation and invasion of glioma cells. UBL7-AS1 was highly expressed in glioma tissues and cells. The overexpression of UBL7-AS1 promotes the cell proliferation and invasion of glioma. UBL7-AS1 can act as a sponge for miR-144-3p in glioma cells. The overexpression of UBL7-AS1 can reverse the inhibition of TMP on proliferation, migration, and invasion of glioma cells. TMP inhibits the proliferation, migration, and invasion of glioma cells by regulating the UBL7-AS1/miR-144-3p pathway.

## 1. Introduction

Gliomas originate in the neuroepithelium [1]. Brain glioma has rich blood vessels, rapidly grows, and easily invades normal brain tissues [2]. Glioma has poor clinical prognosis, high recurrence rate, and resistance to radiotherapy and chemotherapy [3] and is currently the leading cause of cancer-related death worldwide [4–7]. Its occurrence has complex biological characteristics involving a series of pathophysiological changes and alterations in the expression of various genes and signaling pathways [8]. The present clinical treatment effect of glioma is poor [6, 9]. With research progress on the molecular biological characteristics of glioma, the abnormal expression of long noncoding RNA (lncRNA) and its effect on the development of glioma has become a new research hotspot [10, 11].

Tetramethylpyrazine (TMP) was extracted from Chinese traditional medicine *Ligusticumchuanxiong Hort*. TMP has vasodilation and antiplatelet activities [12]. It also has antioxidant and anti-inflammatory effects and can reduce inflammatory injury of endothelial cells induced by lipopolysaccharide or low density lipoprotein [13, 14]. TMP can inhibit tumor growth, invasion, and drug resistance through multiple pathways and multiple targets [15–18]. However, the inhibitory effect and potential mechanism of TMP on glioma cells have not been clarified.

lncRNAs include 5ʹ⁃Cap and 3ʹ⁃Poly (A) domains. Most lncRNAs are transcribed by RNA polymerase II [19] and act as justice or antisense transcripts from intergene regions or other transcripts [20, 21]. lncRNAs are involved in regulating many important human physiological processes, such as chromatin modification, gene imprinting, transcriptional regulation, and posttranscriptional regulation. Moreover, lncRNAs are associated with the occurrence and progression of tumors [22–24]. An abnormal lncRNA expression may be associated with DNA damage, immune escape, and abnormal tumor cell metabolism. lncRNAs may also be closely related to the regulation of epithelial mesenchymal transformation and tumor stem cells in various tumors. Targeting the lncRNA may become a new method for tumor treatment [25]. UBL7-AS1 is abnormally expressed in leukemia [26]; however, its role in glioma has not been reported. The gene sequence of miR-144 is located on chromosome 11, and its expression is downregulated in various cancers [27, 28]. miR-144 can affect the biological function of cancer cells by targeting multiple genes. Han et al. [29] indicated that miR-144 could inhibit the proliferation and migration of ovarian cancer cells by targeting RUNX1. Ren et al. [30] and Ying et al. [31] proposed that miR-144 acts on Pim-1 proto-oncogene (Pim1) and cyclooxygenase-2 genes to inhibit gastric cancer and esophageal squamous cell cancer cells, respectively.

Whether TMP affects the proliferation, migration, and invasion of glioma cells by regulating the UBL7-AS1/miR-144-3p pathway is unknown. In this study, U118MG glioma cells were taken as the research subject to explore the effects of TMP on the proliferation, migration, and invasion of glioma cells. Meanwhile, the regulatory mechanism of TMP on the UBL7-AS1/miR-144-3p pathway was analyzed. This study provides a theoretical basis for revealing the antitumor effects and possible targets of TMP.

## 2. Methods

### 2.1. Cell Culture

Normal human astrocytes (NHAs) and human glioma cell lines A172, T98G, U118MG, and U251 were purchased from the Chinese Academy of Sciences Cell Bank (Shanghai, China). The cells were cultured in the medium of RPMI 1640 (Hyclone) and 10% FBS (Gibco) in a humidified incubator at 37°C with 5%CO_2_. When the degree of cell fusion reached more than 80%, the cells were obtained and used for subsequent experiments.

### 2.2. Cell Transfection

The cells were transfected using lipofectamine 2000 (Invitrogen) reagent following the instructions. has-miR-144-3p mimics was purchased from GenePharma (Shanghai, China). UBL7-AS1 overexpression plasmid pcDNA3.1-UBL7-AS1 and wild-type and mutant UBL7-AS1 reporter gene plasmids (pmirGLO-UBL7-AS1-WT) were constructed in the laboratory. The cells were transfected 48 h later and the subsequent tests were performed.

### 2.3. Fluorescence Quantitative PCR (qRT-PCR)

Total RNA was extracted from the cultured cells treated with the Trizol reagent following the instructions. Reverse transcription was performed using Prime Script TMRT Master Mix. SYBR Green PCR Master Mix was used for qRT-PCR amplification on the ABI7500 Fast Real-Time PCR system. GAPDH and U6 were employed as internal parameters. The relative expression levels were compared by 2^−ΔΔCT^. Sequence information: UBL7-AS1 F: 5ʹ-CTGCTATGGACACAGATGGC-3ʹ, R: 5ʹ-GCCACACACTCTAGGCTCTAC-3ʹ. The upstream primer for GAPDH was 5ʹ-CACAGTCCATGCCATCACTG-3ʹ, and the downstream primer was 5ʹ-ATCTCGCTCCTGGAAGATGG-3ʹ. The relative expression levels of target genes were calculated by the 2^−ΔΔCT^ method, and each sample was detected three times under the same conditions.

### 2.4. CCK-8

CCK-8 assay was used to detect cell proliferation. In brief, 5 × 10^3^ cells per well were inoculated in 96-well plates and treated under different transfection conditions. Each well was added with 20 *μ*L of CCK-8 reagent 72 h after transfection. Absorbance was measured by ELX800 (BioTek) at 450 nm. Cell viability was calculated according to the absorbance value. U118MG and U251 cells were treated with 1000 *μ*M TMP (Dalian Meilun Biotech Co., Ltd, Dalian, China) for 72 h.

### 2.5. Transwell

An invasion experiment was conducted with the Transwell method. A corning Transwell-precoated matrix gel was used for the invasion test. At 24 h after transfection, 3 × 10^4^ cells were suspended in 200 *μ*L of cell suspension and added into a 24-well Transwell compartment. The lower compartment of the 24-well plate was added with 700 *μ*L of medium (containing 10% FBS) and incubated at 37°C for 24 h in the Transwell system. A cotton swab was used to remove cells from the upper surface of the membrane. The cells on the lower surface of the membrane were fixed with 4% formaldehyde and 0.1% crystal violet was stained for 15 min. Five staining cells in the field of vision were randomly selected. Statistical analysis was performed under a fluorescence microscope.

### 2.6. Dual Luciferase Reporter Gene Detection Experiment

The cells were seeded in 96-well plates at 10^4^ seeding density per well. On the second day, 40 nmol/L miR-control or has-miR-144-3p mimic and 0.2 *μ*g of pmirGLO-UBL7-AS1-WT/MUT were co-transfected. This process was repeated for three duplicate holes. After 48 h, 50 *μ*L of the 1 × passive dissolution buffer was added to each well. After incubation on a shaker at room temperature for 20 min, 30 *μ*L of lysis buffer and 100 *μ*L of luciferase buffer were added in sequence. A multifunctional microplate reader was used to detect the firefly luciferase activity and Renilla luciferase activity: luciferase activity = firefly luciferase activity value/Renilla luciferase activity value, statistical analysis. The above steps were applied for the statistical analysis of luciferase activity.

### 2.7. Bioinformatics Analysis

In this study, the expression level of UBL7-AS in glioma and normal brain tissues was analyzed by analyzing the data of glioma in TCGA database. In addition, the correlation between the expression level of UBL7-AS and the prognosis of glioma patients was also analyzed. Data are from GEPIA database (https://gepia.cancer-pku.cn/index.html).

### 2.8. RNA Pull-Down

Biotin-labeled Bio-miR-144-3p and Bio-NC control random sequences were synthesized by TAKARA, and 3ʹ-end biotin labeling was performed. The cells were collected when the degree of syncretic cell growth did not exceed 80%. The transfection reagent used was RNAIMAX. Bio-miR-144-3p and Bio-NC were transfected with 3ʹ-terminal biotin-labeled Bio-miR-144-3p and Bio-NC, respectively, at the final concentration of 10 nM. At 48 h after transfection, the cells were collected for the subsequent detection. Lysed cells and streptavidin-labeled magnetic beads (50 *μ*L for each sample) were also prepared. After incubation for 2 h, the tube with the magnetic beads was placed on the magnetic rack. The supernatant was removed, and the beads were rinsed once with 1 mL of solution buffer, mixed with 500 *μ*L of solution and incubated at 4°C with a rotary mixer. The remaining 50 *μ*L of solution was stored at −80°C for later use. qRT-PCR was performed after RNA isolation.

### 2.9. Statistical Analysis

All experiments were repeated at least three times. SPSS 20.0 statistical software was used for statistical analysis. Measurement data were expressed as mean ± standard deviation. Student's *t*-test was used for comparison between groups. One-way ANOVA followed by Fisher's least significant difference post-hoc test was applied for comparison between the three groups, and *P* < 0.05 was considered statistically significant.

## 3. Results

### 3.1. UBL7-AS1 Is Highly Expressed in Glioma

The expression changes of UBL7-AS1 in tumor tissues and normal brain tissues were first analyzed to study the role of UBL7-AS1 in glioma. The experimental results showed that the UBL7-AS1 expression was higher in glioma tissues than in normal brain tissues (Figure 1(a)). Further survival analysis showed that patients with glioma and high UBL7-AS1 expression had short survival and poor prognosis. To study the role of UBL7-AS1 in glioma, we examined the expression of UBL7-AS1 in human normal glial cells (NHAs) and brain glioma cell lines A172, T98G, U118MG, and U251. The results showed that UBL7-AS1 had the highest expression in U118MG and U251 cells (Figure 1(c), *P* < 0.01). Therefore, U118MG and U251 were selected for subsequent studies. This result suggests that the high UBL7-AS1 expression is related to the occurrence of glioma.

### 3.2. UBL7-AS1 Upregulation Can Promote the Proliferation and Invasion of Glioma Cells

In U251 and U118MG cells, NC was used as a negative control to transfect UBL7-AS1 overexpression plasmid. QRT-PCR results showed that the overexpressed plasmid could upregulate UBL7-AS1 (Figure 2(a), *P* < 0.01). CCK-8 assay revealed that the UBL7-AS1 overexpression promoted the proliferation of U118MG and U251 cells (Figure 2(b), *P* < 0.01). Transwell assay indicated that the invasion ability of U251 and U118MG cells was significantly higher than that of the control group after UBL7-AS1 upregulation (Figure 2(c), *P* < 0.01).

### 3.3. UBL7-AS1 Regulates miR-144-3p Based on ceRNA

lncRNAs may play a promoting role for cancer as ceRNAs. Starbase predicts that UBL7-AS1 may potentially target bind to has-miR-144-3p. The UBL7-AS1 overexpression was predicted to inhibit miR-144-3p in U118MG and U251 cells (Figure 3(a)). However, UBL7-AS1 knockdown upregulated miR-144-3p in U118MG and U251 cells (Figure 3(b)). In addition, the miR-144-3p overexpression inhibited UBL7-AS1. Both genes constituted the regulatory mechanism of ceRNA (Figures 3(c) and 3(d)). Dual luciferase reporter gene assay showed that miR-144-3p could decrease the luciferase activity of pmirGlo-UBL7-AS1-WT but could not change that of pmirGlo-UBL7-AS1-MUT (Figure 3(e), *P* < 0.01). This finding suggests that miR-144-3p can directly bind to UBL7-AS1 by identifying specific sites. RNA pulldown test results showed that the miR-144-3p probe could enrich and bind to UBL7-AS1 (Figure 3(f)).

### 3.4. miR-144-3p Can Reverse the Cancer-Promoting Effect of UBL7-AS1

UBL7-AS1 could regulate miR-144-3p. Hence, their biological roles were further studied. First, changes in the expression level of miR-144-3p after different treatments were detected. The experimental results showed that the UBL7-AS1 overexpression could inhibit miR-144-3p. However, miR-144-3p was upregulated after the transfection of UBL7-AS1 overexpressed plasmid and miR-144-3p mimics (Figures 4(a) and 4(b)). In addition, an interaction between miR-144-3p and UBL7-AS1 in glioma cell growth was determined by CCK-8. The UBL7-AS1 overexpression promoted the growth of U251 and U118MG cells, but this effect was reversed after co-transfection with miR-144-3p and pcDNA3.1-UBL7-AS1 (Figures 4(c) and 4(d), *P* < 0.01). The role of miR-144-3p and UBL7-AS1 in glioma cells was also determined by the Transwell assay. The results showed that the UBL7-AS1 overexpression promoted the invasion of U251 and U118MG cells, but this tumor-promoting effect was inhibited after co-transfection with miR-144-3p and pcDNA3.1-UBL7-AS1 (Figures 4(e) and 4(f), *P* < 0.01).

### 3.5. TMP Inhibits Glioma Cells through the UBL7-AS1/miR-144-3p Pathway

Figure 5 shows the molecular formula of TMP. The results of cell proliferation and invasion experiments showed that TMP inhibited the proliferation and invasion ability of glioma cells (Figures 5(b) and 5(c)). qRT-PCR results showed that compared with the control group, the expression level of UBL7-AS1 in TMP group was significantly decreased (Figure 5(d), *P* < 0.05), while the expression level of miR-144-3p was significantly increased (Figure 5(e), *P* < 0.05). Further experiments showed that the UBL7-AS1 overexpression reversed the effects of TMP on the proliferation and invasion of U118MG cells. Compared with TMP + pcDNA group, the inhibition rate of cell proliferation in TMP + UBL7-AS1 group was decreased (Figure 5(f), *P* < 0.05), and the number of cell invasion was increased (Figure 5(g), *P* < 0.05).

## 4. Discussion

Glioma is the most common primary intracranial tumor, accounting for 81% of malignant brain tumors [8]. This tumor is invasive because of the poor prognosis [32]. Imaging is an effective method for diagnosis and molecular therapy is still the main treatment [33]. This study focuses on a new molecular pathway of glioma development. Evidence shows that the ectopic expression of lncRNA plays an important role in tumor biological processes [34–37].

lncRNAs play a regulatory role as ceRNAs [38, 39]. Lu et al. [40] showed that lncRNA BC032469 promotes the proliferation of gastric cancer cells by upregulating human telomerase reverse transcriptase through miR-1207-5p. Fang et al. [41] reported that lncRNA HNF1A-AS1 promotes the metastasis of colon cancer by regulating the expression of miR-34a/SIRT1/p53 and acting as a ceRNA. However, the potential role of UBL7-AS1 in glioma remains unclear.

This work explored the expression of UBL7-AS1 in glioma cells. The results showed that UBL7-AS1 was highly expressed in glioma cell lines, implying that this gene may be a lncRNA associated with the occurrence of glioma. Interference experiments confirmed that downregulating UBL7-AS1 can inhibit the proliferation, invasion, and migration of glioma cells. In addition, upregulated UBL7-AS1 was associated with the occurrence of glioma. Starbase software analyzed potential miRNAs acted upon by UBL7-AS1. The results showed that miR-144-3p had a high matching degree with UBL7-AS1. Interaction between miR-144-3p and UBL7-AS1 was verified by dual luciferase reporter gene identification and cell activity assay. The results suggested that UBL7-AS1 promoted the growth of glioma cells through miR-144-3p. MiR-144-3p plays as a tumor suppressor in tumors. Chen et al. [42] reported that miR-144-3p could inhibit the proliferation of lung cancer cells, promote apoptosis and autophagy, and play a tumor suppressive role. Song et al. [43] showed that upregulating miR-144-5p could enhance the radiosensitivity of non-small-cell lung cancer cells with radiosensitivity, thus suggesting its tumor suppressive role. Current results revealed that miR-144-3p overexpression could inhibit the migration and invasion ability of glioma cells.

The results of this study showed that the expression level of UBL7-AS1 in glioma cells was significantly decreased after TMP treatment. Further studies showed that inhibition of UBL7-AS1 expression significantly increased the proliferation inhibition rate of glioma cells and significantly reduced the number of invasive cells. These results suggest that TMP may inhibit the development of glioma by inhibiting the UBL7-AS1 expression. The results of this study showed that the expression level of miR-144-3p in glioma cells was significantly increased after TMP treatment. It is speculated that TMP may play an antiglioma role by regulating the UBL7-AS1/miR-144-3p molecular axis. To verify the above speculation, in this study, a UBL7-AS1 overexpressed plasmid was transfected into glioma cells, which were then treated with TMP. The results showed that the proliferation inhibition rate of glioma cells was significantly decreased and TMP inhibited the migration and invasion of glioma cells. These results suggest that TMP can play an antiglioma role by downregulating UBL7-AS1 and upregulating miR-144-3p.

## 5. Conclusion

In conclusion, TMP can inhibit the proliferation, migration, and invasion of glioma cells. Its mechanism is related to the regulation of the UBL7-AS1/miR-144-3p pathway. This will lay a theoretical foundation for further study of TMP antitumor metastasis and its molecular mechanism. This study can also provide a new direction for the development of drugs against glioma metastasis. However, this study only took one glioma cell as the research subject, and subsequent experiments will take multiple glioma cell lines as the research subject to analyze the molecular mechanism of TMP against glioma. At the same time, in vivo experiments and clinical studies are needed to further verify the results.

## Figures and Tables

**Figure 1:** UBL7-AS1 expression in glioma tissues and cell lines. (a) The expression level of UBL7-AS1 in GBM. The data are downloaded from the GEPIA database (https://gepia.cancer-pku.cn/index.html). (b) Prognostic analysis of UBL7-AS1 and glioma patients. The data are downloaded from the GEPIA database (https://gepia.cancer-pku.cn/index.html). (c) UBL7-AS1 is upregulated in glioma cell lines. Data are presented as the mean ± SD. ^*∗*^*P* < 0.05 and ^*∗∗*^*P* < 0.01.

**Figure 2:** Upregulation of UBL7-AS1 promotes the proliferation and invasion of gliomas. (a) qRT-PCR analysis of UBL7-AS1 expression after transfection of NC and UBL7-AS1 into U118MG and U251 cell lines. (b) Measurement of the proliferation ability of glioma cell lines after UBL7-AS1 is upregulated by the CCK-8 method. (c) Detection of the invasion ability of U118MG and U251 glioma cell lines after UBL7-AS1 is upregulated by a transwell experiment. NC : negative control. Data are presented as the mean ± SD. ^*∗∗*^*P* < 0.01.

**Figure 3:** UBL7-AS1 can act as a sponge for miR-144-3p in glioma cells. (a) The expression level detection of the effect of knocking down UBL7-AS1 on miR-144-3p. (b) Detection of the expression level of the effect of overexpression of UBL7-AS1 on miR-144-3p. (c) Detection of transfection efficiency of miR-144-3p mimics. (d) After overexpression of miR-144-3p, UBL7-AS1 expression level detection. (e) Report carrier experiment. (f) RNA pull-down. Data are presented as the mean ± SD. ^*∗∗*^*P* < 0.01.

**Figure 4:** The response experiment proved that the overexpression of miR-144-3p reversed the promotion effect of UBL7-AS1 on glioma. (a) Detection of the expression level of miR-144-3p in U251 cells. (b) Detection of the expression level of miR-144-3p in U118MG cells. (c) CCK-8 detection of the U251 cell proliferation test. (d) CCK-8 detection of theU118MG cell proliferation test. (e) U251 cell invasion experiment after different treatments. (f) U118MG cell invasion experiment after different treatments. Data are presented as the mean ± SD. ^*∗∗*^*P* < 0.01.

**Figure 5:** TMP inhibits glioma cells through the UBL7-AS1/miR-144-3p pathway. (a) Molecular formula of TMP. (b) The CCK-8 method was used to measure the proliferation ability of glioma cell line. (c) Detection of the invasion ability of glioma cell line by a transwell experiment. (d) qRT-PCR analysis of UBL7-AS1 expression after treatment with TMP. (e) qRT-PCR analysis of miR-144-3p expression after treatment with TMP. (f) The CCK-8 method was used to measure the proliferation ability of glioma cell line. (g) Detection of the invasion ability of glioma cell line by a transwell experiment. Data are presented as the mean ± SD. ^*∗*^*P* < 0.05 and ^*∗∗*^*P* < 0.01.

## Data Availability

The data used to support the findings of this study are available from the corresponding author upon request.
